# Light-Weighted Deep Learning Model to Detect Fault in IoT-Based Industrial Equipment

**DOI:** 10.1155/2022/2455259

**Published:** 2022-06-29

**Authors:** Mukesh Soni, Ihtiram Raza Khan, Sameer Basir, Raman Chadha, Arnold C. Alguno, Tapas Bhowmik

**Affiliations:** ^1^Department of CSE, University Centre for Research & Development, Chandigarh University, Mohali, Punjab 140413, India; ^2^Computer Science Department, Jamia Hamdard, Hamdard University, Delhi, India; ^3^Department of Computer System Engineering, University of Engineering and Technology, Peshawar, Pakistan; ^4^Computer Science & Engineering, Chandigarh University, Gharuan, Punjab, India; ^5^Department of Physics, Mindanao State University—Iligan Institute of Technology, Iligan City 9200, Philippines; ^6^Canadian University of Bangladesh, Dhaka, Bangladesh

## Abstract

Industry 4.0, with the widespread use of IoT, is a significant opportunity to improve the reliability of industrial equipment through problem detection. It is difficult to utilize a unified model to depict the working condition of devices in real-world industrial scenarios because of the complex and dynamic relationship between devices. The scope of this research is that it can detect equipment defects and deploys them in a natural production environment. The proposed research is describing an online detection method for system failures based on long short-term memory neural networks. In recent years, deep learning technology has taken over as the primary method for detecting faults. A neural network with a long short-term memory is used to develop an online defect detection model. Feature extraction from sensor data is done using the curve alignment method. Based on long-term memory neural networks, the fault detection model is built (LSTM). In the end, sliding window technology is used to identify and fix the problem: the model's online detection and update. The method's efficacy is demonstrated by experiments based on real data from power plant sensors.

## 1. Introduction

The purpose of equipment failure detection is to help detect equipment failures so as to arrange equipment repair and maintenance and reduce the phenomenon of equipment over-repair. In Industry 4.0, fault detection plays a vital role in reducing production costs in modern industries. Fault detection is mainly used to evaluate the health status of equipment [1]. The online fault detection method plays a crucial role to detect fault in IoT-based industrial equipment. In this method, sliding window technique is used to integrate equipment failure detection and online model updating, enabling the model to react to changes in the condition of the equipment, enhancing accuracy of the model, and decreasing false alarm rate. The retrieved characteristics are input into the defect detection model to determine the model's projected value.

Due to the fast growth of the Internet of Things, numerous sensors are being put on industrial equipment to monitor its health. As a result, a defect detection model may be built using the sensor data obtained to assess the equipment's probable flaws. The usage of IoT provides a great potential to increase the dependability of industrial equipment by detecting problems. The current method of IoT can adjust to changes in the equipment's operational condition and increase the model's detection performance. The limitation of IoT is that due to the complexity of the data models, training is quite costly. With the advancement of deep learning in recent years, defect detection approaches based on deep understanding have gained popularity [2–4], and feature extraction is critical to this strategy. This is because manually selecting reliable sensor data as input characteristics from a large number of sensors is difficult. Additionally, because the model requires a vast quantity of data to learn, it cannot be put directly into the model if we compare the original feature extraction method with the proposed method. The method given in this study reduces the dimension of the feature vector while keeping the original data. It can also accurately judge the equipment's operating position by analyzing the equipment's valuable data.

Numerous academics have employed feature extraction algorithms in recent years to extract relevant characteristics from raw sensor data [5–8]. In high-dimensional data, feature extraction techniques may be used to extract nonredundant variables [9]. It can convert a collection of correlated datasets into a collection of mutually independent characteristics by computing the eigenvectors of the original input's covariance matrix. Previously published work [10] offered a delay correlation-based feature extraction approach for efficiently extracting features from high-dimensional data using delay correlation.

However, in the actual industrial production environment, the equipment is affected by various factors (external environment and self-deterioration), and the sensor data generated by it are also time-varying. The predictive model of the equipment cannot learn all the data at one time. That is to say, models known using historical sensor data have been unable to predict current device state information accurately. For example, large and medium-sized units in thermal power plants are in a high-load state of long-term operation, and equipment deterioration will reduce equipment performance. Using the model trained with historical data will increase the false alarm rate and issue incorrect early warning information to allow professionals to conduct inspections on power plant equipment. Overhaul increases the cost of power plant equipment maintenance.

The model must also react to changes in the operational status of the power plant's equipment over time. As a result, this article presents an online detection approach for equipment failures based on long short-term memory neural networks. Its primary contributions are as follows: a delay-related feature extraction algorithm is used in the data preprocessing stage to further reduce the cost of model training; and the sliding window technology is used to implement equipment fault detection and online model update, allowing the model to adapt to changes in the state of the equipment, thereby improving the model's accuracy and lowering its false alarm rate. The sliding window approach identifies the ongoing detection data stream and updates the model by sensing the device's condition. In this research, the authors have used two types of sliding windows: fixation sliding window and a dynamic sliding window.

The present article has been planned into six sections.  Section 1 describes the introduction of the proposed research.  Section 2 puts light on related work, and the problem analyses are mentioned in Section 3. Online fault detection methods have described in Section 4. The experiment and evaluation has described in Section 5, and finally, Section 6 portrays the conclusion and possible future works based on the proposed framework.

## 2. Related Work

### 2.1. Equipment Fault Diagnosis

Machine learning techniques are the most often used in fault detection, ranging from simple linear discrimination to more complicated logistic regression and neural networks used to problem detection in equipment [9]. The transfer factor analysis approach (TCA) is based on the Gaussian latent factor model for extraction of features, on this basis, developed a linear model for fault identification. This is a way of combining machine learning models in which the accurate output of one model is employed to train the second model to train a higher-precision classifier to meet the goal of defect detection. Gu et al. [11] used the vibration analysis method to obtain user input features for the sensor data collected from wind turbines. It then uses a support vector machine to build a classification model to detect equipment failures. Nayak et al. [12] proposed a transfer factor analysis algorithm (TCA) based on the Gaussian latent factor model for feature extraction, and this basis trained a linear classifier for fault detection. Lang et al. [13] proposed a method of mixing machine learning models, that is, constructing two machine learning models simultaneously, and the correct output of one model is used to train the other machine learning models to train a higher-precision classifier to achieve the purpose of fault detection. The goal of equipment fault detection method is to assist in detecting equipment failures in order to schedule equipment repair and maintenance and prevent the problem of equipment over-repair. This method plays an important role in reducing production costs in modern industries.

Li et al. [14] analyzed the sensor data of the wind turbine with professional knowledge and, after feature extraction, uses the hyperparameter search method to train the support vector machine model to diagnose faults. Finally, Yokouchi and Kondo [15] introduced a single-class SVM model to learn the boundary of the common data space by collecting the equipment's average data and applying it to the fault detection of the equipment.

To a certain extent, the preceding research discusses defect detection, but their approaches cannot be directly applied to predictive maintenance in large-scale companies. This is primarily because the data volume generated by the power plant is enormous and there is a delayed correlation between the data from different sensors, and the operation state of the power plant equipment changes over time, and the above methods are incapable of responding to this change in time. We refresh the model. The model's performance will deteriorate with time.

### 2.2. Online Detection of Equipment Faults

In recent years, an increasing number of researchers have focused on the problem of not being able to learn all failure modes across the equipment's life cycle when training samples are limited or missing, and have presented several solutions. In the absence of fault samples and the difficulty to identify new problems owing to the independence of the training and testing phases, the author [16] presented an anomaly detection and fault diagnosis approach based on online adaptive learning. The technique incorporates classification and clustering algorithms, disrupting the typical mapping between anonymous data and fault kinds. In the testing phase of the AHr detector, samples of known kinds are classified and instances of unknown types are grouped together. The light-weighted deep learning model is different from the traditional deep learning model in term to their performance. The most significant distinction with deep learning and regular machine learning is its effectiveness as information scale expands. Deep learning techniques do not perform well if the information is limited. The author [17] proposed the use of an online sequence extreme learning machine (OS-ELM) for failure identification based on signal reconstruction, recognizing that the existing training set does not adequately reflect all possible conditions encountered during the equipment declaration cycle. OS-ELM possesses a significant capacity for learning, rapid training, and online learning. The implementation of an actual instance indicates that the detection model based on OS-ELM may continually learn and improve detection performance in a developing environment. However, it is still missing a set of decision criteria for when to invoke OS-update ELM's function in response to changing operating conditions. The author [18] suggested a unique hybrid technique for identifying chiller subsystem failures by training on average data and using available failure training data to compensate for the lack of accessible failure training data. The most critical feature variables are chosen using a hybrid feature selection approach. By integrating an extended Kalman filter (EKF) model and a recursive one-class support vector machine, it is integrated into an online classification system (ROSVM). The deployment of an actual example shows that an OS-ELM-based detection model can improve and enhance detection performance and efficiency in a changing environment. The online sequence extreme learning machine (OS-ELM) provides a specific capacity for learning, rapid training, and online learning [19]. However, the approaches outlined above do not take into account sensor datasets with latency correlations and need specialized empirical expertise.

## 3. Problem Analyses

First, the historical data are preprocessed, and the effective feature offline training model is obtained through the delay-related feature extraction algorithm [20]. Then, the online detection of faulty equipment and the online update of the model are realized using a sliding window. Finally, the fault detection model uses the sensor data after feature extraction as the practical input of the model to obtain the predicted value. The method used in this research is more accurate than existing methods. Because the current method can adjust to changes in the equipment's operational condition and increase the model's detection performance, it also analyzes the training effectiveness of different methods in terms of training time. The purpose of fault detection is to accurately judge the equipment's operating status by analyzing the equipment's relevant information. First, the definition of fault detection in this study is given as follows.

Model training using supervised learning, given a set of data *R* = ((*y*_1_, *x*_1_), (*y*_2_, *x*_2_),…, (*y*_*m*_, *x*_*m*_)). *y*_*i*_ is a set of input sensor data vectors, and *x*_*i*_ is the predicted sensor value label during training. We train a neural network model such that

(1) $$\begin{array}{c} N\;\approx \text{Fund}\left(y,x\right). \end{array}$$

Among them, *N* represents the network model, and Fund represents the mapping relationship between *y* and *x* learned by the network model. Given a set of data *y*_*i*_, we output the predicted value *x*_*i*_^∧^ according to the model N and calculate the difference between the expected value and the actual value:

(2) $$\begin{array}{c} e=\left|x_{i}^{\wedge }-x_{i}\right|. \end{array}$$

A threshold *ε* is set for judging the state of the equipment if *e* ≤ *ε*, the equipment is considered regular operation, and vice versa.

But when the equipment runs for some time, the operating state of the equipment may change over time, making the model:

(3) $$\begin{array}{c} N\;\neq \text{Fund}\left(y,x\right). \end{array}$$

The proposed model is used that has been trained with historical data, which can result in a higher percentage of false alarms and erroneous advance warning signals, making it difficult for specialists to conduct audits on power plant equipment. The cost of power plant equipment maintenance rises as a result of overhaul.

The model trained using historical data can no longer accurately describe the running state of the current device. Therefore, at this time, it is necessary to detect the running state of the device and consider using the newly generated sensor data to train the model to update the model parameters to adapt to the current running state of the device.

We use a real case to explain the phenomenon of equipment state change. For example, hundreds of power generation equipment in thermal power plants runs continuously [21]. More than 7,000 sensors are deployed on each generator set to produce real-time sensing data to reflect the operating status of the equipment.

Figure 1 shows the operating principle of the wind and smoke system in a power plant, showing the actual and model-predicted values of the primary fan motor current. In the early stage of equipment operation, a model with better performance has been trained based on historical sensor data. However, as the power generation equipment operates for a long time, it will deteriorate, and the trend of the sensor data generated by it will also change. As a result, the previous model's output is difficult to represent the current state of the equipment. As shown in addition in Figure 1, the system will continuously issue early warning information according to the production of the model and the current data trend, which increases the false alarm rate of the model. At this point, the model itself needs to be updated.

Therefore, when the model predicts the device state, if the model is relearned and updated in time without considering the state change of the device, the device state will be misjudged, resulting in a decrease in the model's accuracy and an increase in the false alarm rate high [22]. Therefore, it is crucial to consider the change of equipment operating state when constructing the fault detection model.

## 4. Online Fault Detection Methods

The structure for the online fault detection model developed in this article is shown in Figure 2. It is broken into three sections: (1) feature extraction for delay correlation: primarily for delay correlation between power generation equipment, extracting features from sensor data, and converting high-dimensional data to low-dimensional data [10]; (2) fault detection model: primarily using long short-term memory neural networks, developing an equipment fault detection model; (3) online fault detection method: primarily using sliding windows, enabling online fault monitoring.

### 4.1. Sliding Window

A sliding window is an algorithm that updates the collected data in real time. The adjacent data are defined as a window. The latest data are added to the sliding window when new data are obtained, and the older data are eliminated. As time goes on, the window continues to incorporate new data and discard the old data, thereby realizing the online detection of faults. In this study, the sliding window consists of a fixed-size FSW (fixation sliding window) and a dynamic sliding window DSW (dynamic sliding window), as shown in Figure 3.

Due to the delay correlation between sensors, the period of FSW is set as Δu, and Δu is the time deviation calculated in the curve alignment algorithm during data preprocessing, which can ensure that in the real-time detection stage, the data in the window can be do alignment and get useful features as input to the model after feature extraction. The period of DSW is *σ*, *σ* is a variable value, and its primary purpose is to save historical data. When the model runs well, we increase the *σ* value, and then, the sliding window can contain more system state areas, making the model prediction more accurate; when the model false alarm rate is higher than the baseline value, we decrease the *σ* value to discard the relatively long history data so that the sliding window only contains recent data for the online update of the model to adapt to the current operating state of the equipment.

### 4.2. Online Detection Method Based on Sliding Window

In the detection process, when the data stream fills the sliding window, data processing starts: the data in the window are extracted and calculated by the curve alignment feature to obtain valuable features, the extracted features are used as the input of the fault detection model to obtain the predicted value of the model, calculate the absolute value of the difference between the predicted value and the measured value of the sensor to determine whether the fault occurs, calculate the false alarm rate of the data in the current sliding window, and the current false alarm rate is compared with the baseline false alarm rate, if it increases, it reduces the size of the sliding window and reacquires data for online model updating; otherwise, we increase the sliding window so that the sliding window can contain more device states.

## 5. Experiment and Evaluation

### 5.1. Experimental Environment and Experimental Data

The experimental environment is a cluster with eight nodes; each node is a machine with an 8-core Intel Xeon (E312xx) CPU, 32 GB memory, 1 GB bandwidth, and Ethernet connection. Each node runs in a virtual machine, using the CentOS6.4 operating system and Java 1.8. With the help of the Spark platform, the Spark Mlib library can be used to run the PCA feature extraction algorithm in a distributed manner.

The data used in the experiments come from accurate sensor data from thermal power plants. Five essential types of equipment in the smoke and wind system were selected, and a total of 290 sensors were deployed on them, and the data generated by the sensors were sampled every 3 minutes. The data collection time was from 00:00:00 on 2018-07-01 to 2020-01-31 at 23:59:59.  Table 1 provides some of the datasets in the experiments. The fault log files are derived from the DCS log files and are used to verify the accuracy of fault detection results.

### 5.2. Experimental Indicators

This article trains a predictive model for defect detection using deep learning techniques and converts it to a binary classification issue by comparing the difference between the anticipated and actual values and a threshold. As a result, there are four possible consequences when a problem is detected. True positive (TP) and true negative (TN) results indicate that the classification was right, but false positive (FP) and false negative (FN) results indicate that the classification was erroneous.

Precision, recall, false positive rate (FPR), F1 score, and receiver operating characteristic (ROC) curves are employed to evaluate experimental outcomes in this research.

### 5.3. Experimental Setup

The fault detection model detects equipment anomalies and deploys them in a natural production environment. For example, we compare our method with the following form for detecting anomalies in power plants.

  R-model (rule model): traditional rule-based anomaly detection methods are based on experience accumulation and implemented rule-based statistical control charts. A fault is found as soon as the sensor data exceed the upper or lower limit.
  P-model (PCA model): input the sensor data after feature extraction by the PCA algorithm into LSTM to detect equipment failure
  SWCP model (sliding window curve registration CA-model): use a sliding window to record the data in the recent period, use the curve to align the data in the window, and then use PCA for feature extraction, input into the model for fault diagnosis, when the false alarm rate is high. At baseline values, the model is updated to fit the current device state.

Both the P-model and SWCP model are neural network models based on LSTM. The LSTM network model used in this study is a fully connected LSTM neural network model, which includes four hidden layers, each with 50 neurons, and its structure is shown in Figure 4. HL*i*: 50 means the *i*th hidden layer, and it has 50 neuron nodes.

Based on the network structure in Figure 4, all weight parameters are uniformly initialized in the range of [−0.08, 0.08]. The model can remember all memories in the initial stage of training. The initial bias value of the LSTM forgetting gate is set to 1.0, and the input gate and the initial value of the output gate are a random floating-point number on the interval [0, 1]. The network was then trained using microbatch stochastic gradient descent with a learning rate of 0.001 and a decay factor of 0.95. The mean squared error is used as the loss function. The model is trained for 50 epochs, and the learning rate is multiplied by a decay factor of 0.95 for each period after ten generations. We choose 80% as the training set and the rest as the test set.

Table 2 provides the dimensions of input feature vectors for different devices. The *L* value in the table represents the data dimension after feature extraction, which is also the dimension of the input vector of the neural network. Based on the training data of the input vector in Table 2 and the experimental environment set in Section 5.1, the initialized LSTM network is trained to obtain the final model parameters, and the effectiveness of the proposed method is verified on the test set.

### 5.4. Experimental Results and Analysis

The findings demonstrate the efficacy of the approach used in this research. This research uses deep learning techniques to develop a model for detection of defects and then transforms it to a binary classification problem by comparing the difference between expected and actual values against a criterion. In this study, each experiment is carried out ten times, and the average value of the ten times results is given in Table 2.

Figure 5 with Table 3 show the accuracy of different methods applied to other devices. The average precision of the rule-based approach was 0.554, and the highest precision was 0.66. The average precision of the P-model is 0.736, the maximum accuracy is 0.79, the average precision of the SWCP model is 0.79, and the utmost precision is 0.82.

Figure 6 and Table 4 show the recall rates of different methods applied on other devices. The rule-based approach has an average recall of 0.488 and a maximum of 0.52. The average memory of the P-model is 0.807 with a maximum of 0.82; the average recall of the SWCP model is 0.862 with a maximum of 0.88.

In addition, for the method proposed in this study, when building the network model, this study tries to reduce the number of hidden layers of the neural network model (3 hidden layers and 45 neurons in each layer), the trained model, and the output prediction results. The average precision is 0.65, and the average recall is 0.74. When the number of hidden layers is increased (6 hidden layers and 60 neurons in each layer), the average accuracy of the output prediction results of the trained model is 0.791 45, and the average recall rate is 0.856 98, which will not improve the prediction. The precision and recall rate of the output is good, but the average training time is 3.4 h.

Figure 7 and Table 5 show the false positive rate of different methods applied on other devices. The rule-based method has an average false positive rate of 0.44 and a minimum of 0.416. The average false positive rate for the P-model approach was 0.157, with a minimum of 0.13. The SWCP model has an average false positive rate of 0.136 and a minimum of 0.118.

Figure 8 and Table 6 show the F1 scores of different methods applied on other devices. For example, the mean F1 score of the P-model process was 0.77 with a maximum of 0.805; the mean F1 score of the SWCP model was 0.82 with a maximum of 0.84.

Since the LSTM model in this study is a binary classification model, the ROC curve is used to verify the classification effect. The curve area of the SWCP model is more significant than that of the P-model and the R-model. The better the classification effect, the better the fault diagnosis effect.

The experimental findings in Figures 5–8 show objectively that predictive maintenance based on deep learning is more successful than traditional rule-based techniques. Additionally, as seen in Figure 7, the SWCP model successfully minimizes the false positive rate, while Figure 8 shows the model's overall performance, demonstrating that the SWCP model has a better score. As a result, it is determined that the strategy presented in this article contributes to the enhancement of feature extraction and model performance in applications.

Additionally, this article analyzes the training effectiveness of various approaches in terms of training time. As shown in Figure 9, we use the same training data as in Section 5.1 to train the model on the cluster set and compare the training times of different models.

The average training time for the P-model is 2.412 h, whereas the average training time for the SWCP model is 2.1 h, as shown in Figure 9 and Table 7. Our technique requires less training time than the P-model. This demonstrates that the feature extraction approach employed in this study is capable of efficiently extracting features from high-dimensional data, hence drastically reducing the quantity of training data and lowering the LSTM neural network's training cost. As a result, the strategy presented in this article aids in the development of a lightweight defect detection model based on LSTM neural networks.

## 6. Conclusion

The online detection method of equipment faults based on the long short-term memory neural network proposed in this study considers the changes of equipment operating status during the online detection phase so that the model can continuously adapt to the equipment running status over time. The light-weighted deep learning has numerous advantages as well as some limitations. As such, due to the complexity of the data structures, training is quite costly. The equipment's predictive model cannot be trained all the data at once, that is, models developed using previous sensor data have failed to reliably anticipate current device status information.

The method in this study adopts the delay-related feature extraction method in the data preprocessing part, which reduces the dimension of the data and reduces the cost of model training; the sliding window technology detects the online detection data stream, and the model is updated by detecting the state of the device. Finally, it is verified by the actual data analysis of the power plant. The approach proposed in this research helps in the creation of a lightweight defect detection model based on LSTM neural networks. The future scope of the lightweight defect detection model method is that it will support in the detection of equipment failures so that equipment repair and maintenance can be handled and the problem of equipment over-repair can be reduced. In addition, proposed research will be helpful in future research studies. The results show the effectiveness of the method in this study: (1) compared with the original feature extraction method, the method in this study further reduces the dimension of the feature vector while ensuring that the original information is included; (2) in the online detection stage of faults, it can adapt to changes in the operating state of the equipment and improve the detection accuracy of the model.

## Figures and Tables

**Figure 1:** Example of sensor flow data for the wind and smoke system [20].

**Figure 2:** Proposed frameworks.

**Figure 3:** Framework of the method in this study.

**Figure 4:** LSTM neural network model structure diagram [12].

**Figure 5:** Accuracy of different methods.

**Figure 6:** Recall of different methods.

**Figure 7:** False positive rate of different methods.

**Figure 8:** F1 scores of different methods.

**Figure 9:** Training time.

**Table 1:** Experimental data table.

Equipment	Number of sensors	Data record	Number of equipment failures
Steam turbine body	111	278400	28
Secondary fan	37	278400	21
Coal mill B	49	278400	18
Primary fan	44	278400	14
Air preheated	49	278400	12

**Table 2:** The input feature vector *L* is the final experimental result.

Equipment	*L* value
Steam turbine body	28
Secondary fan	11
Coal mill B	12
Primary fan	13
Air preheated	13

**Table 3:** Accuracy of different methods.

Serial	Steam turbine body	Secondary fan	Coal mill B	Primary fan	Air preheater
R-model	0.6	0.5	0.55	0.5	0.65
P-model	0.8	0.7	0.8	0.71	0.7
SWCP model	0.8	0.8	0.75	0.8	0.8

**Table 4:** Recall of different methods.

Serial	Steam turbine body	Secondary fan	Coal mill B	Primary fan	Air preheater
R-model	0.49	0.51	0.5	0.45	0.43
P-model	0.78	0.8	0.8	0.83	0.8
SWCP model	0.82	0.82	0.81	0.83	0.85

**Table 5:** False positive rate of different methods.

Serial	Steam turbine body	Secondary fan	Coal mill B	Primary fan	Air preheater
R-model	0.41	0.42	0.43	0.43	0.45
P-model	0.13	0.15	0.12	0.2	0.14
SWCP model	0.11	0.13	0.13	0.15	0.14

**Table 6:** F1 scores of different methods.

Serial	Steam turbine body	Secondary fan	Coal mill B	Primary fan	Air preheater
P-model	0.745	0.743	0.802	0.765	0.761
SWCP model	0.803	0.829	0.803	0.84	0.84

**Table 7:** Training time.

Serial	Steam turbine body	Secondary fan	Coal mill B	Primary fan	Air preheater
P-model	3.4	2	2.52	2.52	1.5
SWCP model	2.5	1.59	2.5	2.5	1.5

## Data Availability

The data used to support this study are available from the corresponding author upon request.
